The article "Osmotic Demyelination Syndrome: Clinical, Neuroimaging Characteristics, and Outcomes in a Series of 18 Cases" was retracted in 2024. Reasons: signs of a paper mill; suspected computer-generated content; unreliable results or conclusions; concerns about the data.

# Osmotic Demyelination Syndrome: Clinical, Neuroimaging Characteristics, and Outcomes in a Series of 18 Cases

**DOI:** 10.1155/2021/9944632

**Published:** 2021-05-28

**Authors:** Xinhuang Lv, Qian Hong, Xiuxiu Lin, Weian Chen, Yuan Tian

**Affiliations:** ^1^Department of Neurology, First Affiliated Hospital of Wenzhou Medical University, Wenzhou, 325000 Zhejiang, China; ^2^Department of Respiratory Medicine, First Affiliated Hospital of Wenzhou Medical University, Wenzhou, 325000 Zhejiang, China; ^3^Department of Hematopathology, First Affiliated Hospital of Wenzhou Medical University, Wenzhou, 325000 Zhejiang, China

## Abstract

**Objective:**

To investigate the etiology, clinical as well as neuroimaging characteristics, and outcomes after proper treatment in a series of 18 patients with osmotic demyelination syndrome.

**Methods:**

Medical records, including video records, of 18 patients with osmotic demyelination syndrome were retrospectively examined. Demographic and clinical information, imaging results, plans of management, and outcomes during the follow-up period were collected and analyzed.

**Results:**

Eighteen patients, including 10 males and 8 females, were included in the present study. The mean age at diagnosis of CNS insult was 47.4 ± 13.3 years (ranged from 30 to 78 years). Etiologies included rapidly corrected hyponatremia (50%), alcoholism (27.8%), and others. Neurological manifestations included encephalopathy (61.1%), dysphonia (50%), extrapyramidal symptoms (38.9%), and seizures (22.2%). Neuroimaging results showed that 6 patients (33.3%) had central pontine myelinolysis, 5 (27.8%) had extrapontine myelinolysis, and 7 (38.9%) had both. After treatment, 12 patients showed improvement and the other 6 did not. Among these patients, those who showed symptoms of encephalopathy had a favorable outcome. The majority of those who presented with mental retardation, seizures, and no other symptoms recovered better than their counterparts who had other symptoms. Nine out of 11 patients with pseudobulbar paralysis and/or extrapyramidal symptoms showed improvement, but the other 2 did not show improvement. Five patients who did not improve after treatment during admission were followed up for 1-3 months with rehabilitation training recommended, and it was found that 3 showed significant improvement after training, and the other 2 did not respond to this training.

**Conclusions:**

Osmotic demyelination syndrome is a complex disease entity due to a variety of etiologies, manifesting with symptoms involving diverse systems of the brain. Early identification and removal/correction of conditions leading to osmotic demyelination syndrome are the key to prevent and/or manage this disease.

## 1. Introduction

Osmotic demyelination syndrome (ODS), including central pontine myelinolysis (CPM) and extrapontine myelinolysis (EPM), is a rare condition and was first described by Adams et al. in 1959 as a noninflammatory, demyelinating condition involving the pons of the hindbrain [1]. In 1962, another 2 studies reported that other brain areas like the basal ganglia, thalamus, cerebral cortex, and the subcortical white matter were also involved in addition to the pons [2, 3]. In the 1970s and 1980s, it was recognized that chronic alcoholism, long-lasting malnutrition, and rapid correction of hyponatremia were the primary causes of ODS, especially when the level of sodium increased by more than 12 mmol/l/d [4].

Although the underlying mechanism of ODS is unclear, it is widely accepted that the pathologic changes observed in ODS were due to compression of fiber tracts by the fluctuating osmotic forces and the subsequent demyelination of these fiber tracts [5].

Clinical manifestations of ODS vary depending on the brain regions afflicted, ranging from symptoms of encephalopathy, pseudobulbar palsy (including dysarthria and dysphagia), to paralysis and extrapyramidal symptoms. The typical radiological findings on MRI are hyperintensities in the central pons and/or other brain regions like the basal ganglia and the thalamus on T2-weighted (T2W) and fluid-attenuated inversion recovery (FLAIR) images and hypointensities on T1-weighted (T1W) images [6–8]. Diffusion-weighted imaging (DWI) also showed increased signal intensity and ADC values [9]. Surprisingly, radiological changes were still present for a period even after clinical improvement was observed.

Currently, the diagnosis of ODS primarily depends on the detailed medical history and imaging findings of suspected patients [7]: (1) a clear history of patients presenting with new neurological symptoms after a rapid increase in the level of serum sodium; (2) characteristic MRI findings include hypointensities on T1-weighted images and hyperintensities on T2-weighted, DWI, proton density-weighted, and FLAIR images. These demyelinated lesions are frequently confined to the central pons and are trident in shape, sparing fiber tracts traveling in the ventrolateral pons, such as the corticospinal tracts.

Though pharmacologic treatment is initiated for patients with ODS immediately after the diagnosis is confirmed, patients do not show consistent improvement as reported by previous studies [1, 10]. Recently, studies suggested that early diagnosis and intensive medical treatment may improve patients' outcomes [9, 11]. Since the 1970s, diverse etiologies have been revealed and treatments for ODS slowly shifted to focus on correcting these conditions apart from correcting patients' symptoms [10]. However, due to the fact that the majority of previous studies were case reports and the underlying conditions were different from each other, no consensus on the prognosis of ODS patients has been reached. In China, a few studies have reported the clinical manifestations of patients with ODS, but only a small number of patients in each study were reported. Here, we presented a large series of 18 patients with ODS in China, summarizing their etiologies, manifestations, neuroimaging findings, treatments, and prognosis after proper management.

## 2. Materials and Methods

### 2.1. Study Participants and Data Collection

Medical records, neuroimaging results, and videotapes of 18 patients with ODS who presented to the First Affiliated Hospital of Wenzhou Medical University from July 1996 to November 2019 were retrospectively reviewed and analyzed.

The diagnosis of ODS was made based on symptoms at admission and additional symptoms during their hospital stay, new hypointensities, or hyperintensities on MR images of different modalities [5]. Diagnostic criteria of ODS were (1) a clear history of patients presenting with new neurological symptoms after a rapid increase in the level of serum sodium; (2) characteristic MRI findings including hypointensities on T1-weighted images and hyperintensities on T2-weighted, DWI, proton density-weighted, and FLAIR images [7]. Demographic information including sex and age, neurological symptoms at presentation, CNS lesions shown on MRI, etiology, locations of new CNS lesions, characteristics of ODS, accompanying neurologic symptoms, and outcomes after treatments were reviewed and extracted. Outcomes were assessed by viewing medical records of patients with ODS and their videos before and after their treatments.

## 3. Results

### 3.1. Demographic Information about Patients with ODS

A total of 18 patients were included in the present study, including 8 males and 10 females with a mean age of 47.4 ± 13.3 years (ranging from 30 to 78 years). Among them, 8 patients showed new neurological symptoms before presenting to our hospital, and the other 10 patients demonstrated new symptoms during their admission (Supplementary Table 1).

### 3.2. Etiologies of Patients with ODS

Eight patients demonstrated new neurological symptoms before arriving at our hospital, and 5 were due to habitual drinking of alcohol, 1 due to uremia, 1 due to myeloma, and 1 due to hypokalemia. The other 10 patients presented new symptoms during their admission. One presented with neurological symptoms after a liver surgery. The other 9 had hyponatremia which was rapidly corrected. As a result, these patients showed neurological deficits. The average level of serum sodium before and after sodium supplementation was 111.2 ± 9.4 mmol/l and 136.1 ± 5.1 mmol/l, respectively, and the median of serum sodium before and after sodium supplementation was 117 mmol/l (in the range of 99-122 mmol/l) and 138 mmol/l (in the range of 127.5-142 mmol/l), respectively. The daily increase in serum sodium exceeded 12 mmol/l. Patient 6 was admitted to our hospital due to hypokalemia (2.8 mmol/l). The most common causes of ODS were the rapidly corrected hyponatremia in (9 patients), followed by alcoholism (5 patients). Three patients had both the rapidly corrected hyponatremia and alcoholism. Other causes included multiple myeloma (1 patient), uremia (1 patient), use of terlipressin (1 patient), hypokalemia (1 patient), post-liver surgery (1 patient), hypernatremia (1 patient), and diabetes insipidus (1 patient) (Table 1).

### 3.3. Neurological Manifestations of Patients with ODS

Clinical manifestations of ODS varied depending on the brain regions involved. The most common one was encephalopathy, which was observed in 11 (61.1%) patients, followed by dysphonia in 9 patients (50%), extrapyramidal symptoms in 7 patients (38.9%), and seizures in 4 patients (22.2%). The most common manifestation of those 9 patients with rapidly corrected hyponatremia was encephalopathy (8/9), followed by severe coma and epilepsy which were observed in 3 patients. Among 5 patients with alcoholism, the most common symptom was dysphonia (4/5), followed by encephalopathy (3/5) and sensory disturbances (3/5) (Supplementary Table 1).

### 3.4. Neuroimaging Data

MRI scan was completed to confirm the diagnosis of ODS for these 18 patients. Among them, 6 showed CPM, evidenced by hyperintensities in the central pons on T2W as well as FLAIR images and hypointensities on T1W; 5 showed EPM involving the basal ganglia and the thalamus; and the other 7 showed both CPM and EPM (Figures 1 and 2). Three out of 5 patients with alcoholism showed CPM. Among 9 patients with their serum sodium rapidly corrected, 8 showed EPM or EPM plus CPM, and 1 showed CPM. The patient with hypokalemia showed CPM. The patient with myeloma and the one with uremia demonstrated CPM, whereas the one treated with terlipressin showed EPM and the one who underwent liver surgery showed CPM and EPM (Figures 1 and 2). The most frequently inflicted brain region was the pons (13/18), followed by the basal ganglia (10/18), the cerebral cortex (6/18), the thalamus, the midbrain, the hippocampus (2/18), and the cerebellum (1/18) (Table 2).

### 3.5. Etiology Oriented Management

The aim of treatment was to remove/correct the conditions that led to ODS. Apart from the specific management plan for patients with concomitant diseases, all of them were managed to sustain their blood volume, to restore levels of electrolytes and the acid-base balance, to provide nutritional support, and to improve their symptoms. For those with rapidly corrected hyponatremia, the speed of supplementing sodium was decreased. For patients with severe symptoms, they were empirically managed with dexamethasone 10 mg once a day for a week. For a patient who was taking terlipressin, this medication was discontinued due to the suspected effect on water and electrolyte disturbance (Supplementary Table 1).

### 3.6. Prognosis

The prognosis of patients with different clinical manifestations was also different. Among these 18 patients with ODS, 12 showed improvement after treatment. Among these 12 patients, 6 completely recovered from ODS. The other 6 did not show significant improvement after treatment, and 1 of them completely failed to respond to the treatment. Patient 4 showed symptoms of respiratory failure and was supported with a ventilator (Table 3, Supplementary Table 1).

In general, patients with symptoms of encephalopathy had a favorable outcome after correcting electrolyte imbalance and supplementing necessary nutrients. The majority of these patients presented only with mental retardation and seizures. These patients recovered better after receiving proper treatment than their counterparts with other symptoms. Among 11 patients with pseudobulbar paralysis and/or extrapyramidal symptoms, 9 showed improvement, and the other 2 did not show significant improvement. Eight of these patients still had mild to moderate neurological deficits.

For patients with pseudobulbar palsy and/or extrapyramidal symptoms, 5 patients were followed up for 1-3 months with their rehabilitation training continued, which included soft palate function training and limb movement-related training. It was found that patients 5, 8, and 12 showed significant improvement in swallowing and speech, whereas patients 13 and 15 did not show significant improvement.

## 4. Discussion

ODS, a rare neurological condition, was poorly understood about its pathogenic mechanism and optimal managements. Though it was first reported in 1959 [1], the majority of available publications about it were case reports. The present study summarized findings from 18 patients with ODS, a large case series study in China, and presented their etiologies, clinical manifestations, neuroimaging results, treatments, and prognosis.

In the present study, it was found that the leading causes were rapidly corrected hyponatremia (50%) and alcoholism (27.8%), followed by other uncommon causes, which is consistent with findings from previous studies [2, 12, 13]. In a study, 292 patients were admitted because of suspected metabolic encephalopathy and 8.56% of them were confirmed ODS patients [5], suggesting that ODS might be closely related to abnormal metabolism. In our study, apart from 6 patients who had ODS after rapidly correcting hyponatremia alone, 5 patients had ODS due to alcoholism (including 3 patients with both the rapidly corrected hyponatremia and alcoholism). Among these alcoholic patients, alcohol might serve as a trigger resulting in vitamin B deficiency, which increases the susceptibility of these patients to demyelinating damage. Furthermore, diagnosing ODS in alcoholic patients is challenging as symptoms of ODS can overlap with alcohol withdrawal. Therefore, extra care should be taken in correcting hyponatremia and in early identification of ODS symptoms in alcoholics [14]. However, a study found that ODS was nearly cured after overcorrecting hyponatremia [15]. Hypokalemia has been reported to be a risk factor of OSD [16]. It was found that 89% of OSD patients who presented with hyponatremia also had hypokalemia [15, 16]. The authors believe that hypokalemia may also increase the susceptibility of nerve fibers to demyelination. In the present study, among the 9 patients who were rapidly corrected for hyponatremia, 6 had serum potassium below 3.5 mmol/l and 1 patient had only hypokalemia during the biochemical examination at the time of onset with a normal level of blood sodium. Specific mechanisms require further research.

The onset of ODS is usually acute and can progress rapidly. Different etiologies lead to different clinical manifestations of ODS. It has been reported that the major neurological symptoms include encephalopathy, parkinsonism, pseudobulbar palsy, and other movement disorder-related symptoms [5, 7, 17]. In our study, encephalopathy (61.1%), dysphonia (50%), extrapyramidal symptoms (38.9%), and seizures (22.2%) were frequently observed, which is similar to findings of previous studies. Due to the fact that the majority of publications reported a small number of patients, predominantly from Caucasian populations, there might be a slight difference in the clinical manifestations between them and Chinese people, which might be confirmed by pooling reports from different ethnic groups.

Neuroimaging is key to the diagnosis of ODS. Based on the location of demyelinating lesions, ODS is divided into CPM and EPM [18]. These two categories of lesions can be observed in the same brain or in different ones. A study reported that 10% of patients with CPM can have concomitant EPM [19]. However, another study reported that CPM plus EPM, CPM alone, and EPM alone accounted for 50%, 30%, and 20%, respectively, of patients with ODS [20]. Among 18 patients with ODS in the present study, 7 (38.9%) had both CPM and EPM, 6 (33.3%) had CPM alone, and 5 (27.8%) had EPM alone. In our study, 3 out of 5 patients with alcoholism had CPM, whereas 8 out of 9 patients with rapidly corrected hyponatremia had EPM or EPM plus CPM. Again, due to the small number of patients studied, the predominance of CPM or EPM cannot be clearly differentiated based on the difference in the underlying causes.

Regarding the brain regions that are commonly inflicted by ODS, it is recognized that the pons in the brainstem is the primary lesion site, followed by the basal ganglia and the thalamus. A study on 58 patients with ODS suggested that the cerebellum and the lateral geniculate body were the most frequently affected extrapontine regions [20]. Another study on 25 patients showed that the pons and the basal ganglia were the most frequently affected regions [5]. Our results are consistent with those of previous reports in that the brainstem, basal ganglia, and the thalamus accounted for 72.2%, 55.6%, and 11.1% of lesion sites, respectively. This might be related to the presence of densely packed fiber tracts in these regions. A rapid increase in osmotic pressure in these regions is more likely to compress these fiber tracts, leading to lesions observed on MR images.

Current treatments for ODS are mainly to remove or correct underlying conditions and to improve symptoms. Acute electrolyte disturbance is fatal under certain circumstances [21]. For all patients, removing or correcting the underlying conditions should be the first step. In general, life-threatening symptoms will be improved after increasing the concentration of serum sodium by 5%. To minimize the risk of developing ODS, serum sodium should not be increased by more than 8-12 meq/l per day. For those who have accompanying risk factors like alcoholism, malnutrition, or hypokalemia in addition to hyponatremia, serum sodium should not be increased by more than 8 meq/l per 24 h [7, 22].

In the present study, 12 out of 18 patients with ODS showed improvement after correcting the underlying conditions, adjusting the speed of supplementing sodium as well as providing nutritional support. When patients were grouped by the time they received treatments, it was found that 2 out of 4 patients who received treatments 24 hours after symptom onset showed improvement during the follow-up period, whereas 10 out of 14 patients who were managed within 24 hours after symptom onset showed improvement and 6 of them completely recovered. This might be explained by the early removal of underlying conditions and consequently halting the progression of ODS. Therefore, early identification of new neurological symptoms and the underlying conditions is key to good outcomes of these patients.

In addition, a relationship between the therapeutic effect and clinical manifestations was observed. For example, patients who showed symptoms of encephalopathy and seizures tended to have better outcomes after treatment than those who had dysarthria and/or extrapyramidal symptoms. This might be related to the extent of brain damage. For patients with severe clinical symptoms, it was suggested that corticosteroid might be effective [5]. In the present study, 2 patients with poor therapeutic response received short-term intravenous administration of 10 mg dexamethasone. One patient showed improvement while the other did not. It is unclear whether this difference is related to the use of corticosteroid or related to the nature and duration of the disease.

Furthermore, rehabilitation training was recommended to patients with unsatisfactory functional recovery. During the follow-up period, 3 out of 5 patients showed improvement in swallowing and speech. This suggests that continued rehabilitation is beneficial to the recovery of patients. Other potential therapeutics such as immunoglobulin injection and plasma exchange are suggested, but further research is required to confirm their usefulness for ODS [23–26].

In conclusion, ODS has diverse etiologies and discrete clinical manifestations as well as neuroimaging characters. Treatments are mainly targeting to correct the underlying conditions and to improve the symptoms. Outcomes are related to various factors. Further research is needed to comprehend this condition.

## Figures and Tables

**Figure 1:** Central pontine myelinolysis: (a) T2 and (b) T2 FLAIR images demonstrating symmetric hyperintensities in the central pons; (c) axial diffusion weighted image; (d) ADC map demonstrating restricted diffusion changes in the central pons; (e) sagittal T1 image demonstrating hypointensities in the pons.

**Figure 2:** Extrapontine myelinolysis with central pontine myelinolysis: (a, b) axial diffusion-weighted images demonstrating restricted diffusion in the cerebral cortex and the basal ganglia; (c) T1 and (d) ADC map showing hypointensities in the basal ganglia; (e) T2 image demonstrating symmetric hyperintensities in the basal ganglia; (f) T2 FLAIR image demonstrating symmetric hyperintensities in the central pons.

**Table 1:** Etiologies of ODS.

Etiologies	*N* (%) *n* = 18
Hyponatremia	9 (50.0)
Alcoholism	5 (27.8)
Multiple myeloma	1 (5.6)
Uremia	1 (5.6)
Terlipressin used	1 (5.6)
Hypokalemia	1 (5.6)
After general anesthesia	1 (5.6)
Hypernatremia	1 (5.6)
Diabetes insipidus	1 (5.6)

**Table 2:** Distribution of lesions in the brain.

Lesion site (s)	*N* (%) *n* = 18
Pons	13 (55.6)
Basal ganglia	10 (55.6)
Cerebral cortex	6 (33.3)
Midbrain	2 (11.1)
Thalamus	2 (11.1)
Hippocampus	2 (11.1)
Cerebellum	1 (5.6)

**Table 3:** Clinical characters of participants.

Patient	Age (y)	Sex	Treatment	MMSE (before)	MMSE (after)	Water swallowing test (before)	Water swallowing test (after)	GCS (before)	GCS (after)	Water swallowing test (after rehab)
1	54	M	Symptomatic treatment	29						

2	30	M	Symptomatic treatment	29						

3	53	F	Symptomatic treatment	18	29					

4	78	F	Symptomatic treatment+dexamethasone 10 mg	Not cooperative	Not cooperative	Not cooperative		6	10	

5	30	M	Symptomatic treatment+dexamethasone 10 mg			4	3			2

6	38	F	Symptomatic treatment	20	29	1	1			

7	52	M	Symptomatic treatment	17	28	4	2			

8	47	F	Symptomatic treatment	20	29	4	3			2

9	34	F	Symptomatic treatment	15	26	4	3			

10	61	M	Symptomatic treatment							

11	60	M	Symptomatic treatment			3	2			

12	26	F	Symptomatic treatment			3	2			1

13	55	M	Symptomatic treatment			4	3			3

14	40	M	Symptomatic treatment	16	27	2	2			2

15	39	M	Symptomatic treatment	20	29					

16	58	F	Symptomatic treatment	18	29					

17	49	M	Symptomatic treatment	18	28	3	2			

18	50	F	Symptomatic treatment	19	29					

## Data Availability

Data are available from the corresponding author upon reasonable request.

## Supplementary Materials

Supplementary Materials Supplementary Table 1: clinicoradiologic information of ODS patients.
